The article "A Data Augmentation Method for Prohibited Item X-Ray Pseudocolor Images in X-Ray Security Inspection Based on Wasserstein Generative Adversarial Network and Spatial-and-Channel Attention Block" was published in 2022. Journal: Comput Intell Neurosci.

# A Data Augmentation Method for Prohibited Item X-Ray Pseudocolor Images in X-Ray Security Inspection Based on Wasserstein Generative Adversarial Network and Spatial-and-Channel Attention Block

**DOI:** 10.1155/2022/8172466

**Published:** 2022-03-18

**Authors:** Dongming Liu, Jianchang Liu, Peixin Yuan, Feng Yu

**Affiliations:** ^1^College of Information Science and Engineering, Northeastern University, Shenyang 110819, China; ^2^State Key Laboratory of Synthetical Automation for Process Industries, Northeastern University, Shenyang 110819, China; ^3^School of Mechanical Engineering and Automation, Northeastern University, Shenyang 110819, China

## Abstract

For public security and crime prevention, the detection of prohibited items in X-ray security inspection based on deep learning has attracted widespread attention. However, the pseudocolor image dataset is scarce due to security, which brings an enormous challenge to the detection of prohibited items in X-ray security inspection. In this paper, a data augmentation method for prohibited item X-ray pseudocolor images in X-ray security inspection is proposed. Firstly, we design a framework of our method to achieve the dataset augmentation using the datasets with and without prohibited items. Secondly, in the framework, we design a spatial-and-channel attention block and a new base block to compose our X-ray Wasserstein generative adversarial network model with gradient penalty. The model directly generates high-quality dual-energy X-ray data instead of pseudocolor images. Thirdly, we design a composite strategy to composite the generated and real dual-energy X-ray data with background data into a new X-ray pseudocolor image, which can simulate the real overlapping relationship among items. Finally, two object detection models with and without our data augmentation method are applied to verify the effectiveness of our method. The experimental results demonstrate that our method can achieve the data augmentation for prohibited item X-ray pseudocolor images in X-ray security inspection effectively.

## 1. Introduction

With the frequent population flow, people carry more and more items in the baggage and the types of prohibited items have become increasingly abundant. In order to ensure public security, the research studies on the detection method of prohibited items are significant. Currently, X-ray inspection technology has been widely used in the security inspection of public places, reducing criminal behavior effectively. In the process of security inspection, security inspectors need to determine whether there are prohibited items in baggage through the X-ray images. In some special situations, such as the traffic rush hours, the frequency of baggage passing is greatly increased, which requires security inspectors to complete the inspection in a very short time. In addition, there is still no unified standard for the training of security inspectors, and the accuracy of inspection depends on the experience and working status of security inspectors. For these reasons, the accuracy of manual detection methods cannot be guaranteed [1]. Accordingly, a fast and effective automatic detection method of prohibited items for X-ray security inspection is significant.

The detection method of prohibited items has been developed for many years. In the early stage, the automatic detection method of prohibited items usually used different feature extraction algorithms to extract the features of prohibited items and then classified the extracted features. These feature extraction methods included scale-invariant feature transform (SIFT), Haar-like features (Haar), bag of visual words (BOW), histogram of oriented gradients (HOG), and so on [2]. Based on these feature extraction methods, researchers proposed some detection methods of prohibited items. In the case of the single-energy X-ray image, Turcsany et al. [3] proposed a method based on BOW for detecting firearms using a dual-view approach. In [4], a method using visual vocabulary and an occurrence structure was proposed to detect three different prohibited items. In addition, an approach called adaptive sparse representation (XASR+) [5] was proposed to recognize items automatically in cases with less constrained conditions including contrast variations, pose variations, image size variations, and focal distance variations. In the case of the dual-energy X-ray image, Riffo and Mery [6] proposed an active X-ray testing framework that is able to find an adequate view of the object item to detect razor blades in different cases. The applicability of BOW methods in X-ray image classification and retrieval was discussed in [7]. In practical applications, the performance of these automatic detection methods based on manual features cannot meet the requirements due to the wide variety of items, occlusion, noise, clutter, and other reasons.

In recent years, the convolutional neural networks (CNNs) have been widely used in image analysis and processing. Methods based on deep learning have achieved great success in many computer vision tasks [8–10]. A CNN-based classification algorithm was proposed in [9], after which CNN-based classifiers have received wide attention in the field of computer vision. These methods based on the CNN have achieved satisfactory results in image classification [11], object detection [12], target segmentation [13], etc. For the object detection methods based on the CNN, the methods are mainly divided into two classifications. One is the two-stage method, such as R-CNN [12], Fast R-CNN [14], Faster R-CNN [15], R-FCN [16], and FPN [17]. These methods first generate a set of candidate region suggestions and then classify, filter, and refine the candidate region suggestions to achieve object detection. The other is the one-stage method, such as YOLO [18–21] and SSD [22]. These methods predict the classification and bounding box directly from a single convolutional network. Such methods have a faster detection speed, but the accuracy is lower than that of the two-stage methods. Both of them have achieved success in the object detection of natural optical images and have been applied in various fields [23–25].

Compared with natural optical images, X-ray pseudocolor images are quite different in several aspects. Natural optical images are formed by the light reflection, while X-ray pseudocolor images are formed by irradiating the objects with X-ray, which loses a lot of information about the surface of objects [26]. In addition, X-ray pseudocolor images consist of shadows from overlapping transparent layers. The transparency of the pseudocolor image is determined by the material density along the X-ray path and different materials will appear in different colors. The overlap between objects also makes the same object appear in different colors, and high-density objects (e.g., thick metal) can obscure other overlapping objects [27]. These phenomena make the research on object detection of X-ray images difficult. In [28], Mery et al. used transfer learning to classify three kinds of prohibited items based on the X-ray grayscale images, and the experimental results showed that the method is effective. In [29], Akcay et al. compared a BoVW approach with a CNN approach, and the experiments showed that the methods based on the CNN outperform the BoVW methods. In [30], the researchers proposed a method using deep convolutional neural networks to detect objects in X-ray security inspection. The method adopted a specific data enhancement technique, feature enhancement blocks, and multiscale fusion regions of interest. Most of the previous research studies for X-ray security inspection used transfer learning based on the ImageNet dataset. However, the direct adoption of the pretrained networks limits the adjustment of the network structure for X-ray pseudocolor images and may reduce the detection performance.

In addition, the method based on deep learning requires a large amount of data. Nevertheless, the X-ray pseudocolor image dataset is scarce and the color definition of X-ray pseudocolor images varies from company to company, which presents an enormous challenge to the object detection method of prohibited items for X-ray security inspection. There are two methods to solve this problem. One is to collect sufficient X-ray images containing the prohibited items with various poses and scales, which requires huge costs. The other is data augmentation. Using data augmentation methods can improve the generalization ability of the methods based on deep learning. Data augmentation methods include rotation, translation, scaling, etc. However, these methods have limited performance gains for the methods based on deep learning. In the last few years, the generative adversarial network (GAN) has achieved considerable success in image generation [31]. To improve the quality of the generated images, some models based on GAN have been proposed, such as the CGAN [32], the Cycle GAN [33], and the WGAN-GP [34]. Recently, some data augmentation methods based on the GAN have been used for X-ray image datasets. In [35], Yang et al. proposed a method of prohibited item X-ray pseudocolor image generation using the GAN. Their generated X-ray pseudocolor images only contain one single prohibited item and the image quality and diversity are not ideal. In [36], Zhu et al. proposed a method based on Cycle GAN to transform the item natural images into X-ray pseudocolor images. These methods used the methods based on GAN to directly generate prohibited item X-ray pseudocolor images and then replaced the target area of the real background X-ray pseudocolor image with the generated images. It is worth noting that these methods cannot show the real overlapping relationship among items. This also resulted in the fact that the final composite X-ray pseudocolor images are not ideal.

To generate more realistic and higher-quality X-ray pseudocolor images, we propose an effective data augmentation method for prohibited item X-ray pseudocolor images in X-ray security inspection (DA-PIX). The main contributions of the method are as follows. Firstly, we design the framework of the DA-PIX to achieve the dataset augmentation using the datasets with and without prohibited items. Secondly, based on the WGAN-GP, we design a spatial-and-channel attention block (SCAB) and a new base block to compose our X-ray Wasserstein generative adversarial network model (SCAB-XWGAN-GP). The model directly generates high-quality dual-energy X-ray data instead of X-ray pseudocolor images. Thirdly, in order to generate more realistic X-ray pseudocolor images, we design a composite strategy based on the absorption law of X-ray to composite the generated and real dual-energy X-ray data with background data into a new more realistic X-ray pseudocolor image, which can simulate the real overlapping relationship among items.

The rest of the paper is organized as follows.  Section 2 describes the dataset creation. In Section 3, the proposed method is described.  Section 4 presents the experiments and results. Finally, Section 5 concludes the paper and discusses some directions for future work.

## 2. Dataset Creation

The dual-energy X-ray method has been widely used in X-ray security inspection systems. The method realizes the material classification of the detected objects by measuring the difference of attenuation coefficient of different materials under high-energy and low-energy X-ray. The low-energy and high-energy data are converted into an X-ray pseudocolor image by a lookup table to facilitate the interpretation of the detected objects, and the lookup table can be obtained through calibration [37]. In order to clearly distinguish the material of the detected object, orange represents the organic matter, green represents the mixture matter, and blue represents the inorganic matter in the X-ray pseudocolor image.  Figure 1 shows the imaging process of the X-ray pseudocolor image.

The dual-energy X-ray security inspection equipment was provided by Shenyang DT Inspection Equipment Co., Ltd., China. The X-ray tube voltage is 140 kV. The X-ray tube current is 0.75 mA. The value range of the dual-energy X-ray data is normalized to 0–15200. The size of each data is 600 × 600 × 2. Our X-ray dataset is divided into two parts. One is the X-ray prohibited item dataset (XD-P). The XD-P is collected in the simulated situation. To establish the XD-P, different baggage with the random prohibited items is packed and sent into the security inspection equipment. The XD-P consists of 8,000 dual-energy X-ray data and corresponding X-ray pseudocolor images. The prohibited items include brass knuckles, firecrackers, guns, hammers, knives, lighters, metal bottles, pliers, and scissors. The other is the X-ray security item dataset (XD-S). The data in the XD-S are the basic data for the data augmentation. The data in XD-S were collected from the real subway security inspection. The XD-S consists of 10,000 dual-energy X-ray data and corresponding X-ray pseudocolor images without prohibited items. Some X-ray pseudocolor images of the dual-energy X-ray data used in this paper are shown in Figure 2.

## 3. DA-PIX Method

The dataset plays an important role in the object detection methods based on deep learning. Due to the security, the dataset is scarce. In order to augment the dataset and improve the robustness of the method, some methods based on the GAN are proposed. However, these methods are limited for our dataset because these methods cannot show the real overlapping relationship between the generated prohibited items and the background. This also results in the fact that the final composite X-ray pseudocolor images are not ideal. Accordingly, we propose an effective data augmentation method DA-PIX for prohibited item X-ray pseudocolor images in X-ray security inspection. Firstly, we design the framework of the DA-PIX. Secondly, we design the SCAB-XWGAN-GP model that directly generates high-quality dual-energy X-ray data instead of X-ray pseudocolor images. Thirdly, we design a composite strategy to composite the generated and real dual-energy X-ray data with background data into a new more realistic X-ray pseudocolor image.

### 3.1. The Framework of DA-PIX

To obtain more ideal composite X-ray pseudocolor images and improve the robustness of the detection method, we design the DA-PIX. The framework of the DA-PIX is shown in Figure 3. First, the SCAB-XWGAN-GP model is trained using a training dataset extracted manually from the XD-P. Second, the real dual-energy X-ray data of prohibited items and the generated dual-energy X-ray data of prohibited items using the SCAB-XWGAN-GP model are combined into a dataset for the composite strategy. Third, using the secure background dual-energy X-ray data from the XD-S and the foreground dual-energy X-ray data of prohibited items from the dataset for the composite dual-energy X-ray data, new composite dual-energy X-ray data can be obtained through the composite strategy. Then, the composite dual-energy X-ray data can be converted into an X-ray pseudocolor image by a lookup table. The composite images can more realistically simulate the actual situation. Finally, we can obtain the final augmented dataset.

### 3.2. SCAB-XWGAN-GP Model

Some methods based on GAN are applied to generate prohibited item X-ray pseudocolor images. A typical GAN model is composed of a generator and a discriminator. The architecture of the GAN model is shown in Figure 4. The generator is trained to generate the new data from random noise. The discriminator is trained to distinguish between the real data and the generated data.

However, these methods mainly focus on directly generating the X-ray pseudocolor images of prohibited items and cannot show the real overlapping relationship among items. Hence, we need to generate high-quality dual-energy X-ray data instead of X-ray pseudocolor images, which allows our next composite strategy to composite more realistic and higher-quality X-ray pseudocolor images. For the methods based on GAN, most models use upsampling + convolution or transposed convolution. Meanwhile, the X-ray prohibited items dataset is sparse and the training of the methods based on the GAN is challenging, which would result in the methods overfitting or collapse. In order to generate higher-quality prohibited item dual-energy X-ray data, we design the SCAB-XWGAN-GP model. In our model, we use the WGAN-GP as the basis and the dual-energy X-ray data as the generated object. Meanwhile, we design a new base block to compose the generator. The new base block can effectively improve the quality of the generated images and reduce the training difficulty of the discriminator and the generator.

The structure of the base block is shown in Figure 5. In the base block, we employ the convolutional layer and the PixelShuffle in the subpixel convolution [38] to achieve upsampling. The PixelShuffle can rearrange the elements of a *H* × *W* × *C* · *r*^2^ feature map to a feature map of shape *r* · *H* × *r* · *W* × *C*. After that, we use a residual block containing convolutional layers with 3 × 3 kernels to optimize the quality and detail of the generated data. In the process, in order to improve the fitting ability of the block and reduce the training difficulty, we use the ParametricRelu (Prelu) [39] as the activation function.

In addition, to generate more realistic dual-energy X-ray data, we design the SCAB based on the spatial-and-channel squeeze-and-excitation [40] block to fit our SCAB-XWGAN-GP model. The SCAB can make the details of data generated by the generator more realistic. Moreover, it can make the discriminator ignore less meaningful information and focus on more meaningful information. The architecture of the SCAB is shown in Figure 6. Given an input *X* ∈ *R*^*H*×*W*×*C*^, we can get the calibrated output $\tilde{X}\in R^{H\times W\times C}$. The SCAB is divided into the spatial and channel branches.

For the channel branch, *X* can be expressed as *X*=[*x*_1_, *x*_2_,…, *x*_*i*_,…, *x*_*C*_], where *x*_*i*_ ∈ *R*^*H*×*W*^. First, the global average pooling and the global max pooling are used to generate two 1 × 1 × *C* feature maps  *S*_*a*_=[*S*_*a*1_, *S*_*a*2_,…, *S*_*aC*_] and *S*_*m*_=[*S*_*m*1_, *S*_*m*2_,…, *S*_*mC*_] to express *X* in general. Second, the channel-wise dependencies $\tilde{S}$ can be obtained using fully connected (FC) layers and nonlinearity layers. The process can be expressed as

(1) $$\begin{array}{c} \tilde{S}=\varphi \left(W_{a2}\sigma \left(W_{a1}S_{a}\right)+W_{m2}\sigma \left(W_{m1}S_{m}\right)\right), \end{array}$$

where  *φ* is the sigmoid function, *σ* represents the Relu activation function, **W**_*a*1_, **W**_*m*1_ ∈ *R*^*C*/*R*×*C*^,  **W**_*a*2_, **W**_*m*2_ ∈ *R*^*C*×*C*/*r*^ are the weights of the fully connected layers, and *r* is a ratio parameter. Third, the recalibrated feature map of the channels ${\tilde{X}}_{c}$ can be obtained by

(2) $$\begin{array}{c} {\tilde{X}}_{c}=\text{Scale}\left(\tilde{S},X\right)=\left[{\tilde{s}}_{1}x_{1},{\tilde{s}}_{2}x_{2},\ldots ,{\tilde{s}}_{C}x_{C}\right], \end{array}$$

where Scale(·) refers to channel-wise multiplication between the scalar $\tilde{S}$ and the input *X*.

For the spatial branch, *X* can be expressed as *X*=[*x*_1,1_, *x*_1,2_,…, *x*_*i*,*j*_,…, *x*_*H*,*W*_], where *x*_*i*,*j*_ ∈ *R*^1×1×*C*^. The spatial-wise dependencies *O* can be extracted using 1 × 1 convolution layer and the nonlinearity layers. The process can be expressed as

(3) $$\begin{array}{c} O=\varphi \left(\sigma \left(W_{c}X\right)\right), \end{array}$$

where **W**_*c*_ ∈ *R*^1×1×*C*×1^ is the weight of the 1 × 1 convolution layer. Then, the recalibrated feature map of the spatial can be obtained by

(4) $$\begin{array}{c} {\tilde{X}}_{s}=\text{Scale}\left(\tilde{S},X\right)=\left[{\tilde{s}}_{1,1}x_{1,1},{\tilde{s}}_{1,2}x_{1,2},\ldots ,{\tilde{s}}_{H,W}x_{H,W}\right]. \end{array}$$

After obtaining the recalibrated feature maps, the final calibrated output recalibrated feature map $\tilde{X}$ can be obtained by

(5) $$\begin{array}{c} \tilde{X}=X+{\tilde{X}}_{c}+{\tilde{X}}_{s}. \end{array}$$

Based on the base block and the SCAB, we design the SCAB-XWGAN-GP model. The architecture of the SCAB-XWGAN-GP model is shown in Figure 7. In the generator, six base blocks and one SCAB are concatenated to generate 256 × 256 data and the upsampling multiplier for each base block is 2. It is worth noting that the PixelShuffle requires four times the number of channels on its upper layer, which leads to a dramatic increase in computation and the number of parameters. Therefore, we limit the maximum number of channels of the base block to 256. It also means that the number of convolutional kernels per convolutional layer is at most 1024. Finally, we can obtain the generated dual-energy X-ray data through a convolution + tanh block. In the discriminator, the real and fake data are used as input data, and then the feature extraction is performed by six convolution + Prelu blocks and one SCAB. Finally, the predicted results are output through the fully connected layer.

For our SCAB-XWGAN-GP model, we use the same training method and the loss function as the WGAN-GP. The loss function *L* of the SCAB-XWGAN-GP model can be defined as

(6) $$\begin{array}{c} L=E\left[D\left(G\left(z\right)\right)\right]-E\left[D\left(x\right)\right]+\lambda \cdot E\left[{\left(\nabla_{\hat{x}}D{\left(\hat{x}\right)}_{2}-1\right)}^{2}\right], \end{array}$$

where *G* is the generator, *D* is the discriminator, *z* is the random noise vector, *λ* is the penalty coefficient, and $\hat{x}$ is the gradient penalty object sampled from the sample space of the generated data and the real data uniformly, $\hat{x}=\varepsilon z+\left(1-\varepsilon \right)G\left(z\right)$, where *ε* ∈ [0,1].

### 3.3. The Composite Strategy

Through manual collection and the SCAB-XWGAN-GP model, we can obtain a large amount of dual-energy X-ray data for the prohibited items. For compositing the ideal X-ray pseudocolor image, we design the composite strategy based on the absorption law of X-ray. Based on the exponential law of photon radiation attenuation, the energy flux density after passage through the object with the thickness of *d* can be expressed as

(7) $$\begin{array}{c} \varphi =\varphi_{0}e^{-\sigma \;d}, \end{array}$$

where *φ*_0_ is the incident energy flux density and *σ* is the attenuation coefficient. If X-ray radiation passes through  *n* different objects, the energy flux density after passage through the objects can be expressed as

(8) $$\begin{array}{c} \varphi =\varphi_{0}e^{\left(-\sum_{i=1}^{n}\sigma_{i}d_{i}\right)}, \end{array}$$

where *i* = 1, 2,…, *n*. The gray value of a pixel can be linearly modeled as [37]

(9) $$\begin{array}{c} D=A\cdot \varphi +B, \end{array}$$

where *A* and *B* are constant parameters of the model. Since the composite strategies for the high and low energies are same, we take single energy as an example. Define the gray value of the foreground object (*D*_fore _) and the gray value of background object (*D*_back _) as

(10) $$\begin{array}{c} D_{\text{fore }}=A\cdot \varphi_{\text{fore }}+B=A\cdot \varphi_{0}e^{-\sigma_{\text{fore }}d_{\text{fore }}}+B, \end{array}$$

(11) $$\begin{array}{c} D_{\text{back }}=A\cdot \varphi_{\text{back }}+B=A\cdot \varphi_{0}e^{-\sigma_{\text{back }}d_{\text{back }}}+B, \end{array}$$

where *σ*_fore _ and *σ*_back _ represent the attenuation coefficient of *D*_fore _ and *D*_back _ and *d*_fore _ and *d*_back _ represent the thickness of *D*_fore _ and *I*_back _. From (8), the energy flux density of the composite data *φ*_*c*_ can be modeled as

(12) $$\begin{array}{c} \varphi_{c}=\varphi_{0}e^{-\sigma_{\text{fore }}d_{\text{fore }}-\sigma_{\text{back }}d_{\text{a}}}. \end{array}$$

The gray value of the composite data *D*_*c*_ can be expressed as

(13) $$\begin{array}{c} D_{c}=A\cdot \varphi_{c}+B=A\cdot \varphi_{0}e^{-\sigma_{\text{fore }}d_{\text{fore }}}e^{-\sigma_{\text{back }}d_{\text{back }}}+B. \end{array}$$

From (10), (11), and (13), we can obtain

(14) $$\begin{array}{c} \frac{D_{c}-B}{K}=\frac{D_{\text{fore }}-B}{K}\cdot \frac{D_{\text{back }}-B}{K}, \end{array}$$

where *K* is the constant and it can be obtained using a calibration approach [37]. From (14), we can obtain the gray value of the composite data as follows:

(15) $$\begin{array}{c} D_{c}=\frac{\left(D_{\text{fore }}-B\right)\cdot \left(D_{\text{back }}-B\right)}{K}+B. \end{array}$$

We can obtain a composite X-ray pseudocolor image using equation (15) and a lookup table. The details of the composite process are shown in Figure 8. Two random dual-energy X-ray data *D*_fore _ and *D*_back _ are selected (*D*_back _ belongs to the XD-S and *D*_fore _ belongs to the dataset for the composite images). Then, we randomly select the composite position *P* and generate the composite matrix *Mark*. *Mark* is a two-valued matrix of zeros and ones, which is obtained from *D*_fore _ by binarization. Finally, the composite image can be obtained by

(16) $$\begin{array}{c} I_{c}=\text{Lookup}\left(D_{\text{back }}\cdot \left(1-\text{Mark}\right)+C\left(D_{\text{back }},D_{\text{fore }},P,\text{Mark}\right)\right), \end{array}$$

where Lookup(·) represents the conversion of dual-energy X-ray data to X-ray pseudocolor images and *C*(·) indicates the composite operation of *D*_back _ and *D*_fore _ at position *P* using (15).

To demonstrate the superiority of our composite strategy, we show the original X-ray pseudocolor image and the composite X-ray pseudocolor images using different methods in Figure 9. The traditional method uses the foreground to replace the target area of the background. From Figure 9, we can find that the composite X-ray pseudocolor image using our composite strategy can simulate the real overlapping relationship between the prohibited item and the background compared to the traditional method, which makes the composite X-ray pseudocolor image more realistic.

In addition, our composite strategy can not only realize the composite of the single prohibited item and the safety images but also realize the composite of the multiple prohibited items and safety images or images containing prohibited items. Some composite X-ray pseudocolor images are shown in Figure 10. From Figure 10, we can find that the composite X-ray pseudocolor images using our method can simulate the real situation for the single prohibited item and multiple prohibited items. The composite X-ray pseudocolor images using our composite strategy can increase the diversity of our dataset.

Utilizing our composite strategy, we can randomly select the real and generated foreground objects to combine with the data in XD-S into an augmented dataset. By controlling the selection of the foreground objects and the composite position, we can easily control the position of objects in the augmented dataset and achieve a balance in the number of each object. Using the method, we can obtain a nearly infinite augmented dataset.

## 4. Experiments and Results

In this section, we first test our SCAB-XWGAN-GP model. Then, to verify the effectiveness of our DA-PIX, we design a comparative experiment to evaluate the performance of our method. The experiments are run on a GPU system with the following specifications: Intel Core i9-10900k CPU, 64 GB RAM, and NVIDIA GeForce GTX 3090 GPU.

### 4.1. Evaluation Criteria

For evaluating the generated X-ray pseudocolor images, the Fréchet inception distance (FID) [41] is used. The FID is a comprehensive metric that has been shown to be more consistent with human assessments in assessing the realism and variability of the generated samples. We can obtain the FID by calculating the Wasserstein-2 distance between the generated X-ray pseudocolor images and the real X-ray pseudocolor images in the feature space of the Inception-v3 network. Lower FID value means that the distance between the generated data and the real data distribution is closer and the model works better.

For evaluating the performance of the object detection model with and without our DA-PIX, average precision (*AP*) and mean average precision (*mAP*) are used. AP can be calculated as

(17) AP=111∑Re∈0,0.1,0.2,……,1maxR˜e:R˜e≥RePrR˜e,

where *Pr* is the precision (*Pr*=*TP*/*TP*+*FP*),  *Re* is the recall (*Re*=*TP*/*TP*+*FN*), *TP* is the number of true-positive samples, *FP* is the number of false-positive samples, *FN* is the number of false-negative samples, and *Pr*(*Re*) is the measured precision at recall *Re*. Subsequently, *mAP* can be defined as

(18) $$\begin{array}{c} mAP=\frac{1}{K}\sum_{k=1}^{K}AP_{k}. \end{array}$$

### 4.2. Results and Discussion

In order to better verify the effectiveness of our SCAB-XWGAN-GP model, we trained the DCGAN model and the WGAN-GP model to compare them with our model. For the training dataset used by the generative models, first we extracted the object data from the labeled XD-P by labeling the extracted data manually. Second, we kept the target data unchanged and replaced the background with 15200 by manual labeling. Third, we filled these data into a square with the maximum value of the width and height of the data and resized them to 256 × 256 × 2 using the bilinear interpolation. Finally, these dual-energy X-ray data formed the training dataset used by the generative models. The adaptive moment estimation (Adam) optimization algorithm was used. The batch size was 32, the penalty coefficient *λ* was 10, and the learning rate of the generator and discriminator was 0.0002 and 0.0001, respectively. The update ratio of generator and discriminator was 5 for our model and the WGAN-GP model. For the DCGAN model, the update ratio of generator and discriminator was 1. It is worth noting that the generated data by these models are dual-energy X-ray data, and these data are converted into the X-ray pseudocolor images by a lookup table. Some X-ray pseudocolor images generated by these models are shown in Figure 11.

From Figure 11, it can be found that the generated X-ray pseudocolor images by the DCGAN have a lot of noise, the images appear to have severe distortion, and the detailed information is blurred. Meanwhile, for the brass knuckle and plier, the DCGAN showed pattern collapse. For the WGAN-GP, the quality of the generated X-ray pseudocolor images has improved, but there is still noise and distortion in the images, the detailed information is still blurred, and the visual quality is poor. Compared with the methods, although there is still a little noise and minor deformation in the generated X-ray pseudocolor images, the quality of the X-ray pseudocolor images generated using our SCAB-XWGAN-GP is significantly improved.

In addition, to objectively evaluate our method, we compared the methods quantitatively using the FID score. The FID scores of these models are shown in Table 1. From Table 1, we can find that our method has the lowest FID score. This means that our model can better approximate the distribution of the real dual-energy X-ray data of the prohibited items.

Then, to verify the effectiveness of our DA-PIX, we trained the object detection models with and without our DA-PIX. We employed the YOLOV4-tiny model [21] as the object detection model. We randomly divided the XD-P into the training dataset and the testing dataset. The training dataset contained 7200 X-ray pseudocolor images and the test dataset contained 800 X-ray pseudocolor images. Our DA-PIX was used to augment the training dataset. In this process, first, we manually cropped the generated dual-energy X-ray data and resized them to their real size. Second, we combined these dual-energy X-ray data with the real dual-energy X-ray data extracted from the XD-P to form the dataset for the composite strategy. Third, we used the composite strategy to composite the new X-ray pseudocolor images with the data in the XD-S as the backgrounds. These composite X-ray pseudocolor images contained 2–7 prohibited items in each image. The augmented training dataset contained 17,200 X-ray pseudocolor images. After augmenting the dataset, we trained the YOLOV4-tiny model on the training dataset and the augmented training dataset, respectively. The stochastic gradient descent with momentum (SGDM) was used. The batch size was 16, the initial learning rate with warm-up was 0.001, and the momentum was 0.9. The detection results are shown in Table 2.

From Table 2, we can find that the *mAP* of the YOLOV4-tiny model trained by the augmented training dataset is higher than that of the YOLOV4-tiny model trained by the original training dataset, with an increase of 9.25%. Moreover, the AP of each prohibited item has been enhanced using our method. It means that our DA-PIX method can effectively improve the performance of the detection model for prohibited item X-ray pseudocolor images in X-ray security inspection. In addition, the YOLOV4-tiny model is a lightweight detection model, and we believe that the *mAP* will be further improved under more complex detection models.

## 5. Conclusion

In this paper, an effective data augmentation method for prohibited item X-ray pseudocolor images in X-ray security inspection is proposed. The innovation is mainly reflected in three major aspects. First, we design the framework of our DA-PIX to achieve dataset augmentation using the datasets with and without prohibited items. Second, in order to generate high-quality dual-energy X-ray data, a SCAB-XWGAN-GP model is designed based on the SCAB and a new base block. Third, a composite strategy based on the absorption law of X-ray is proposed to composite a new X-ray pseudocolor image, which can simulate the real overlapping relationship among items. Two YOLOV4-tiny models with and without our DA-PIX are trained to verify the effectiveness of our method. The experimental results demonstrate that our DA-PIX can effectively improve the mAP of the YOLOV4-tiny model. Therefore, our DA-PIX is effective for the data augmentation of prohibited item X-ray pseudocolor images in X-ray security inspection.

In future work, we will focus on designing effective detection models for the detection of prohibited item in X-ray security inspection.

## Figures and Tables

**Figure 1:** The imaging process of the X-ray pseudocolor image.

**Figure 2:** Some samples of our dataset. (a) Some samples of the XD-P. (b) Some samples of the XD-S.

**Figure 3:** The framework of the DA-PIX.

**Figure 4:** The architecture of the GAN model.

**Figure 5:** The structure of the base block.

**Figure 6:** The architecture of the SCAB.

**Figure 7:** The architecture of the SCAB-XWGAN-GP (the number under each block represents the size of the data after passing through that block).

**Figure 8:** The composite process.

**Figure 9:** The original X-ray pseudocolor image and the composite X-ray pseudocolor images using different methods. (a) The original X-ray pseudocolor image. (b) The composite X-ray pseudocolor image using our composite strategy. (c) The composite X-ray pseudocolor image using the traditional method.

**Figure 10:** Some composite X-ray pseudocolor images. (a) The original X-ray pseudocolor image. (b–h) The composite X-ray pseudocolor images.

**Figure 11:** Some X-ray pseudocolor images generated by different models. (a) The X-ray pseudocolor images generated by the DCGAN. (b) The X-ray pseudocolor images generated by the WGAN-GP. (c) The X-ray pseudocolor images generated by the SCAB-XWGAN-GP.

**Table 1:** The FID scores of different models.

Items	WGAN-GP	DCGAN	SCAB-XWGAN-GP
Brass knuckle	185.3	143.7	**103.2.**
Firecracker	16.3	18.7	**13.8**
Gun	73.1	121.7	**18.47**
Hammer	32.6	41.8	**19.2**
Knife	25.8	32.3	**9.4**
Lighter	106.9	108.6	**78.3**
Metal bottle	45.2	48.6	**41.4**
Plier	43.8	45.6	**27.2**
Scissors	44.5	48.4	**22.4**

**Table 2:** The detection results.

Items	YOLOV4-tiny + the original training dataset	YOLOV4-tiny + the augmented training dataset
Brass knuckle	88.75%	**95.76%**
Firecracker	86.63%	**92.88%**
Gun	86.80%	**93.84%**
Hammer	67.81%	**80.59%**
Knife	74.20%	**80.58%**
Lighter	86.69%	**94.81%**
Mental bottle	93.17%	**96.23%**
Plier	89.77%	**90.11%**
Scissors	72.79%	**87.06%**
mAP	82.96%	**90.21%**

## Data Availability

The dataset used to support the findings of this study was supplied by Shenyang DT Inspection Equipment Co., Ltd., China, under license and the dataset involving security cannot be shared.
